# Highway Traffic Flow Prediction Model Construction Based on the Gray Theory and BP Neural Network

**DOI:** 10.1155/2022/1120491

**Published:** 2022-07-12

**Authors:** Zaiyang Jiang

**Affiliations:** Constrution Project Office of Wuchang Lalin River Section of Tieke Expressway, Harbin, Heilongjiang 150001, China

## Abstract

The short-term traffic flow prediction and modeling of highways are the core content and important foundation of highway management decision-making support systems. It is of great significance to improving the level of highway management. Based on the macrodynamic traffic flow model, this article establishes a method for establishing a highway traffic flow prediction model based on the BP neural network theory and gray theory. We collected and carry out modeling and prediction of highway traffic flow data near a certain station. It is learned from the prediction results that the traffic flow prediction model based on the BP neural network and gray theory has a high degree of reliability.

## 1. Introduction

With the rapid development of urban transportation, the traffic management department tries to strengthen the mastering of the dynamic characteristics of the traffic network by obtaining real-time traffic information and providing decision-making support for urban traffic management [1–3]. Real-time traffic information provides possible control and induction strategies for the development of traffic management departments. In traffic management, traffic information is the basis of various traffic applications. The deployment of intelligent transportation equipment can help achieve this goal. The ring coil detector is a widely used piece of equipment in the fields of traffic monitoring and communication, and it is also a reliable and efficient way to obtain the dynamics and complexity of urban traffic systems [4–6].

The highway is one of the important features of the development of transportation in modern countries. In the mid-1950s, Western developed countries recovered from the weak economic state after World War II and entered a period of economic sustainable growth and social modernization. Highway transportation demand has continued to increase, and railway transportation demand has relatively decreased. With the continuous improvement of national income levels, the ownership of private cars in developed countries has continued to rise, and cars have become the main passenger tool [7–9]. There are problems in which highway transportation capacity lags behind traffic growth. The construction of ordinary highways cannot significantly improve the timeliness and reliability of automobile transportation [10, 11].

The construction of highways is an inevitable choice to improve highway transportation capacity and make transportation adaptable to the needs of economic development. In the stage of industrialization to mature development, the construction of highways on a large scale has become the common law of transportation development in various countries [12, 13]. Many economically rejuvenated countries also began to build highways in the 1960s and 1970s after developed countries, which also produced huge transportation benefits and socio-economic efficiency. At present, more than 80 countries (regions) around the world have highways, and the mileage of highways has reached more than 220,000 kilometers. The number of highways in the United States, Australia, China, Germany, France, Italy, Japan, and other countries is at the forefront [14, 15].

The highway in China started at the end of the 1980s and has gone through the starting phase of construction from the end of the 1980s to 1997 and the rapid development stage from 1998 to the present. According to the “National Highway Network Plan,” China plans to build a highway network consisting of 7 capitals, 9 north-south longitudinal lines and 18 east-west horizontal lines in about 30 years.

However, while the highway network expands rapidly, the daily operation and management of highways begin to encounter more and more problems. The first is traffic congestion and traffic accidents. The traffic flow status depends on the transportation of traffic participants, with randomness and uncertainty. Traffic flow based on real-time data analysis, considering the randomness of traffic flow time and space, according to the traffic flow data of several periods in the past, can be used to predict the traffic flow estimation value within several periods of time.

As the process of traffic flow changes is a real-time, nonlinear, high-dimensional, nonsmooth random process, as the statistical period is shortened, the randomness and uncertainty of traffic flow changes are getting stronger and stronger. The change in traffic flow is not only related to the traffic exchanges in the past few periods of this section but also affected by factors such as the traffic flow and weather changes, traffic affairs, and the traffic environment. Basic parameter data of traffic flow, such as traffic, average speed, density, and share, can be obtained through various traffic flow information collection equipment. In these data, the data that reflect changes in traffic flow time mainly include the traffic parameters and historical average of this data collection point in the past. Data that reflect changes in traffic flow spaces mainly include the upstream and downstream of this data collection point. The problem to solve the traffic flow prediction is how to from the traffic flow from various traffic flow information collection equipment from various influencing factors.

The specific method of studying can be divided into two types: parameter and nonparameter methods. The parameter method believes that the task of prediction of traffic flow is to assume that there is a formulating function relationship between the input and the output. It can be found through historical data that can make the theoretical output and actual traffic through historical data. A set of parameters with the smallest errors between flow data and then use the models to predict the future traffic flow. For example, the classic self-regression moving average method has the advantages of fast calculation speed and high accuracy. However, with the development of computer technology, the advantages of the fast calculation speed of the ARIMA method are no longer prominent [16–18]. Therefore, the attention of the ARIMA method in the past ten years has been reduced, but when the data is sufficient, the seasonal Arima method is better than the nonparameter regression method. Therefore, the improvement of the method still has not stopped, such as considering the multipoint Arima method. On the other hand, the nonparameter method does not pursue the format of *F* but to find the rules from historical data through some data mining and artificial intelligence methods to form a mapping of input-output. A large amount of historical data is required to ensure the accuracy of the model, and the prediction accuracy is seriously dependent on the universality of the “laws” obtained. The nonparameter method is the research hotspot of the short-term prediction method in recent years.

Based on the actual traffic flow observation, the classic road traffic flow theory divides traffic flow into two categories: free flow and crowded flow. However, by analyzing the measured data for a long time, some researchers further divided squeezed flow into wide movement blockage and synchronization flow. Wide movement is blocked, which is a moving structure where vehicles stop or almost stop. The blocked downstream wave surface spreads to the upstream at a characteristic speed of 15 km/h. In contrast, the downstream wave surface of the synchronous flow is usually fixed at the transportation bottleneck, and the flow of the synchronous flow is much larger than the flow of the wide movement, sometimes even equivalent to the free flow.

The neural network is the earliest nonparameter prediction method. The classic BP neural network can fit the fitting of any form by adjusting the weight of the node, so it is adopted by a large number of studies. Subsequently, some more complex neural networks were also used, such as radial base networks and object-oriented networks. Neural networks are also often used with other algorithms, such as algorithms with Bayesian, combined with Kalman filter algorithms and genetic algorithms. Similar to neural networks, the latest nonparameter prediction method supports the vector machine, which can achieve a good prediction effect.

Based on the macrodynamic traffic flow model, this article establishes a method for establishing a highway traffic flow prediction model based on the BP neural network theory and gray theory. We collected and carried out modeling and prediction of highway traffic flow data near a certain station. It is learned from the prediction results that the traffic flow prediction model based on the BP neural network and gray theory has a high degree of reliability.

## 2. Methods and Theories

### 2.1. BP Neural Network Overview

The artificial neural is a complex nonlinear dynamic system composed of a large number of neurons with a certain topology structure. Because neural networks have the ability to approach any nonlinear mapping through learning, the neural network is applied to nonlinear mapping to nonlinear mapping, and the neural network is applied to non-linear mapping to nonlinearly. The modeling and identification of the linear system cannot be limited by the nonlinear model, which is convenient for the implementation algorithm and the modeling of the complex system.

The working principle of artificial neural networks is similar to the human nervous system, one of which is the most commonly used called BP neural network. The BP neural network is also called an error reverse propagation neural network. It was proposed by Rumelhart and McClelland in 1986. It is a multilayer front-to-neural network. BP neural network has great advantages in nonlinear mapping, self-learning, adaptive, fault-tolerant, etc., and it has been widely used in many areas. The BP neural network is an algorithm for nonlinear function problems. The BP neural network is generally multilayered, mainly divided into three layers of the input layer, hidden layer, and output layer. This is as shown in Figure 1.

It can be seen from Figure 1 that the various layers of the BP neural network are composed of multiple neurons, and the two adjacent layers are connected to each other, but there is no connection between neurons located in the same layer. Its training process consists of two parts: the positive transmission of information and the reverse propagation of errors. When spreading forward, the sample is transmitted layer by layer along the network sequence, and the output value is finally obtained in the output layer. The final value and threshold of the layer are finally approaching the expected value.

The core of the neural network lies in the design of the network structure, which focuses on the number of network layers and the number of nodes of each layer. The theory has proven that increasing the number of network layers can further reduce errors and improve accuracy, but at the same time, it will also make the network complicated, reduce real-time, and increase the training time of the network; the accuracy of the error can be improved, and the observation and adjustment of its training effect are easier than the increase in the number of layers. Therefore, it is generally necessary to give priority to increasing the number of hidden neurons. For the input layer and output layer of the neuron network, you need to study the problems of solving in the instance and the specific representation method to determine the number of neurons.

The traffic model adopted herein is shown in Figure 2. According to the figure, the 6 data amounts of Q1–Q6 are used as the input layer, the number of hidden neurons is 36, and the hidden layer nodes in the article are taken to be 12 in this article.

### 2.2. Gray Theory

Since Professor Deng Julong in China first proposed the theory of gray system control problems in 1982, after more than thirty years of development, this theory has become an emerging marginal discipline, which has become increasingly widely used. The gray system is defined as a known system with some information. It is between white and black. It can only establish a corresponding model for part of the system. Therefore, the structure of the gray system is not completely clear, the factors are relatively incompletely clear, and the mechanism of its role is also incomplete. Due to the complexity of the system composition, the relationship between parallel, constraints, and redundant association between components is very difficult to accurately establish a system equipment state prediction model which can greatly reduce the difficulty of system modeling and meet the requirements for prediction accuracy.

The gray system modeling is based on the weakening of the randomness of the original information, the establishment of a gray “module,” and the use of a difference transforms the time sequence into a differential equation. The use of this model to analyze the system in the system can reflect the nature of the changes in the system's internal mechanism, which can be used to predict control. This is a model that uses insufficient information to establish information as much as possible, and it is also a way to give full play to the role of white information. It is a method of establishing a differential division equation with discrete data. There are mainly accumulation and reduction. Generally, in the case of the numbers, the randomness of the data will gradually weaken with accumulation, and the regularity of the data will be improved. This is as shown in Figure 3.

## 3. Results and Discussion

The data use a section of the highway in Jiangsu Province on January 1, 2021, to a certain number of traffic vehicle charging data at some sites. The purpose is to predict the traffic of one of the stations. The middle station is extracted from the database as the research object. The traffic data of the day and the changes in the traffic in a short period of time are shown in Figures 4 and 5.

From Figure 4, it can be analyzed that the changes in traffic flow throughout the day go through the following stages: traffic flow in the early morning, trough period; morning traffic flow, climbing period; noon traffic, flat peak period; afternoon traffic, peak period; and evening traffic flow decrease. Combined with Figures 4 and 5, the peak of the traffic flow is during 10-11, the short-term traffic changes are very ups and downs, but the overall maintenance is about 10 vehicles per minute. Once again, the changing trend of vehicle traffic changes in nearby sites and comparison with the site discovered that the ups and downs of vehicles near the site are similar, and there is a correlation effect of the changes in vehicle flow between the vehicles between the stations in a short period of time. To this end, this article adopts the above traffic flow prediction model to perform traffic forecasts for the site in a short period of time. This model is simpler than other macrodynamic vehicle traffic models. The corresponding prediction results can also reflect the traffic situation within the current area of the nearby site.

This article starts the simulation prediction for the vehicle flow of the vehicle traffic from 10 to 11 o'clock during the day. During the training, 60 sets of data are trained during the 10-11 period, and 10 sets of data in the next ten minutes are predicted. The change of the traffic training error of 10-11 is shown in Figure 6.

Figure 7 is a control diagram of the simulation result of traffic speed and actual data. The real line is actual traffic data, and the result of the output of the neural network is available. From Figure 7, it can be seen that the further training adjustment of neural networks can reduce errors, so the basic characteristics of traffic integrated based on gray-based and BP neural network models can be well described.

## 4. Conclusion

1. This article simplifies it on the basis of studying the macrodynamic traffic flow model and analyzes the traffic flow of a certain site with changes in time to forecast the highway traffic flow.
2. It is learned from the prediction results that the prediction model of the gray theory and BP neural network traffic flow prediction model has a high degree of reliability. The simplified traffic flow model is more accurate, and the prediction results can also be comprehensively described in a certain space for the certain space of the site.
3. In the prediction of traffic flow, the consideration is not comprehensive, and other factors such as weather and road conditions should be examined to achieve the fusion prediction of polysource data. At the same time, the algorithm is essentially an inspiration. It also needs to be optimized in terms of calculation efficiency and calculation speed to overcome the problem of too long running.

## Figures and Tables

**Figure 1:** BP neural network structure diagram.

**Figure 2:** Traffic flow prediction model.

**Figure 3:** Gray system modeling.

**Figure 4:** The daily vehicle flow of the reference station.

**Figure 5:** The changes of the one-hour car flow of the reference station.

**Figure 6:** Prediction of sample results' comparative analysis.

**Figure 7:** Transport density comparison.

## Data Availability

The figures used to support the findings of this study are included within the article.
